# Correlation Analysis of DNA Methylation in the von Willebrand Factor Promoter Region and the Risk of Unexplained Recurrent Hemophilia: Systematic Review and Meta-Analysis

This article has been retracted.

**DOI:** 10.1155/2022/3977289

**Published:** 2022-06-03

**Authors:** Jing Dong, Jie Li, Ling Yang, Qiuhong Kong, Zhirong Zhang, Hong Zhang

**Affiliations:** The Second Affiliated Hospital of Shandong First Medical University, No. 366 Taishan Street, Tai'an, Shandong 271000, China

## Abstract

This study systematically reviewed the effect of DNA methylation in the promoter region of the coagulation factor vWF gene on the risk of unexplained recurrent hemophilia. PubMed, Medline, Web of Science, and other computers were used to search the database, and the statistical randomized controlled trials of coagulation factor vWF in the risk analysis of unknown recurrent hemophilia were collected. The Cochrane systematic evaluation method was used to evaluate the quality of the included kinds of literature, and Revman5 software was used to sort out and analyze the kinds of literature. Meta-analysis showed that there was a statistical difference between the experimental group and the control group in case fatality rate (OR = 1.76, 95% CI (1.29, 2.39), *P*=0.0003, *I*^2^ = 0%, *Z* = 3.58), adverse events (OR = 2.38, 95% CI (1.65, 3.45), *P* < 0.00001, *I*^2^ = 0%, *Z* = 4.60), incidence of joint hemorrhage (OR = 2.52, 95% CI (1.62, 3.91), *P* < 0.00001, *I*^2^ = 0%, *Z* = 4.12), incidence of subcutaneous stasis (OR = 1.76, 95% CI (1.26, 2.45), *P*=0.0009, *I*^2^ = 5%, *Z* = 3.33), and hematoma volume (OR = 1.78, 95% CI (1.32, 2.40), *P*=0.0001, *I*^2^ = 23%, *Z* = 3.80). DNA methylation in the promoter region of the coagulation factor vWF gene was significantly associated with the risk of unexplained recurrent hemophilia. Whether demethylation can improve the bleeding index of patients with recurrent hemophilia remains to be further explored.

## 1. Introduction

Hemophilia is a group of sexually co-recessive hemorrhagic diseases, which is clinically divided into hemophilia *A* (coagulation factor VIII (FVIII) defect) and hemophilia *B* (coagulation factor IX (FIX) defect), caused by *F* VIII and F IX gene mutations, respectively [1]. In the male population, the incidence of hemophilia *A* and hemophilia *B* is about 1/5 000 and 1/25000, respectively. Hemophilia *A* accounts for 80% to 85% of all male patients with hemophilia, hemophilia B accounts for 15% to 20%, and hemophilia in women is extremely rare. von Willebrand factor (vWF) is a polymeric glycoprotein produced mainly by vascular endothelial cells and is a risk factor for assessing the status of bleeding and thrombosis [2–4]. Under high shear forces, vWF is involved in platelet adhesion and aggregation, leading to thrombosis [5]. vWF gene or any other gene abnormality in the pathogenesis of von Willebrand factor. The incidence of vWF is about 1% [6]. In addition, von Willebrand disease is a common clinical autosomal hereditary hemorrhagic disease, which is caused by the reduction of abnormal function of the vWF. Most hereditary diseases are dominant, and a few are recessive. The incidence is about 1/1000. Clinical manifestations are mainly bleeding of different degrees, such as nasal bleeding, gingival bleeding, skin ecchymosis, bleeding after skin abrasion, excessive menstrual blood volume, postpartum bleeding, and postoperative bleeding [7].

vWF is a hereditary hemorrhagic disorder caused by a deficiency of vWF or abnormal function. Most vWFs are autosomal dominant, and a few are autosomal recessive (AR). According to the pathogenesis and phenotype of vWF, there are three types: type 1 refers to reduced vWF content, but normal function. In this type, the level of vWF: AG, vWF: RCO, and vWF decreased, resulting in a decrease of factor VIII activity, accounting for about 60% of all vWF types, and the bleeding was more serious than that of type I. Type 2 can be divided into four subtypes: 2*A*, 2*B*, 2*M*, and 2*N*. Type IIN is the vWF gene and VIII binding site mutation, FVIII affinity, and hemophilia *A*. Type III is vWF, and the level of FVIII is 5% ∼ 10%. Homozygous or double gene abnormalities may occur in each region of the vWF gene, resulting in the clinical manifestation of severe bleeding. The vWF gene is located at the top of the short arm of chromosome 12 (12p13.3), and the cDNA of vWF generates a primary transcript of 2813 amino acids containing a 22-amino acid signal peptide, a 741-amino acid propeptide (vWFAg: II), and a mature unit of 2050 amino acids. The types of mutations in vWF genes include insertion or deletion mutations, nonsense mutations, splice site mutations, missense mutations, and promoter mutations, with missense mutations being the most common [8]. The main pathogenesis of vWF is vWF gene mutation, and vWF gene detection can help vWF typing and differential diagnosis.

But there are still about 50% of patients with unknown causes, unable to target the cause of treatment and plaguing patients. Studies have shown that screening for thrombotic genes is effective in preventing unexplained recurrent abortions [9]. Coagulation factor vWF is a serine protease synthesized by the liver and plays an important role in fibrinolysis and coagulation. Recent studies have shown that spontaneous abortion is associated with the clotting factor vWF, but its mechanism remains unclear. Epigenetics plays an important role in the regulation of gene expression and genotype characteristics. DNA methylation is an important component of epigenetics and plays an important role in cell differentiation and embryo development [10]. Therefore, this study conducted a meta-analysis to explore the relationship between DNA methylation in the promoter region of the coagulation factor vWF gene and the incidence of recurrent hemophilia of unknown cause.

## 2. Materials and Methods

### 2.1. Search Strategy

The Cochrane Library, PubMed, CNKI, EMBASE, and Wanfang databases were searched by the computer until November 2021. Search the Chinese version of these medical words and keywords and determine the search terms, including “VON Willebrand factor portal hypertension” and “vWF Portal Hypertension”. In order to improve the recall rate, a retrospective search was carried out from the references of relevant literature studies, and all published literature studies meeting the requirements were retrieved (Figure 1).

### 2.2. Literature Inclusion Criteria

1. The retrieval language was English, the retrieval deadline was February 2022, and the study type was a randomized controlled study
2. Patients diagnosed with hemophilia
3. Serum coagulation factor vWF was measured in all subjects
4. The contents included in the literature should be related to the relationship between the antigen concentration of von Willebrand factor and hemophilia
5. The results of serum or plasma coagulation factor vWF were detected within 24 days after admission, and the ELISA method was used to detect vWF antigen level
6. The original data directly or indirectly provide mean and standard deviation or OR value and 95% CI

### 2.3. Literature Exclusion Criteria

1. The experimental design was nonrandomized controlled literature
2. For the two kinds of literature with the same data, the one published for the first time was regarded
3. Literature that cannot provide valid data for analysis
4. The second published literature shall be subject to the highest level of the journal

### 2.4. Data Extraction

Search according to the retrieval strategy described above. In the retrieval process, the initial screening of the literature was carried out according to the title, and the literature that did not meet the inclusion criteria was screened out according to the title and language of the literature. Further screening was carried out by reading the abstract part of the literature after preliminary screening, and the literature studies that met the requirements were kept temporarily. Finally, the literature that will be included in this meta-analysis will be determined by carefully reading the full text of the literature and combining the inclusion and exclusion criteria.

### 2.5. Literature Quality Assessment

Quality Assessment of Diagnostic Accuracy Studies (QUADAS) is a tool for evaluating the quality of literature. It contains 14 evaluation criteria and is used to evaluate the accuracy of diagnostic tests. Each criterion was evaluated by “yes,” “no,” and “unclear”. “Yes” means meeting this standard, “no” means not meeting or not mentioned, and partially meeting or cannot obtain exact information from the literature is regarded as “unclear.”

### 2.6. Bias Analysis

The heterogeneity test, also known as the homogeneity test of statistics, aims to check whether the results of each independent study have the same value. Commonly used measurement methods are the *Q* test and the *I*^2^ test. The level of the *Q* test is usually set as *P*=0.10, that is, heterogeneity exists between studies when *P*=0.10. The value range of the *I*^2^ test is defined as 0–100%. When *I*^2^ < 50%, heterogeneity is acceptable. On the basis of the heterogeneity test, appropriate methods were selected for statistical analysis of the combined effect size. When the heterogeneity is not obvious (*I*^2^ < 50%), the fixed-effect model can be used to estimate the combined effect size. When heterogeneity is obvious (*I*^2^ > 50%), the random-effect model was selected. The commonly used effect size indicators in this study include the following: (1) continuous variable data include weighted mean difference (WMD) and standardized mean difference (SMD) and (2) relative risk (RR), odds ratio (OR), and risk difference (RD) were the effect indexes of dichotomous data. In this paper, the main indicators of combined effect size are odds ratio (OR) and standardized mean difference (SMD), as shown in Figures 2 and 3.

## 3. Results

### 3.1. Literature Retrieval Results and Included Research Characteristics

A total of 800 literature studies on the relationship between vWF antigen level and hemophilia were searched and screened. Finally, 12 literature studies were included [11–22], including 7 literature studies with mean and standard deviation. There were 463 patients in the case group and 265 in the control group. There were 5 literature studies with OR value and a 95% CI, including 799 patients in the case group and 1716 patients in the control group. The screening was conducted in strict accordance with the preestablished inclusion criteria, through preliminary screening and full-text screening, and repeated, non-case-control studies and literature that did not meet the inclusion criteria were excluded. Finally, the selected literature studies are published literature studies. The literature screening process was made according to the statistical software Review Manager 5.2, as shown in Table 1.

### 3.2. Case Fatality Rate

Review Manager 5.2, a statistical software specialized for meta-analysis, was used to extract and summarize the data, and the analysis statistics were used. For WMD and 95% CI, the *Q* test was first used in the heterogeneity test of included studies. Vascular pseudo-Willebrand factor antigen concentration in the case group and control group was used to compare the results of the analysis. First of all, heterogeneity inspection into the results of the study does not exist between heterogeneity and meta-analysis uses the fixed-effect model. The result shows that the case group vascular pseudo-Willebrand factor antigen concentration was higher than the control group. Obviously, the difference was statistically significant, so there was a statistical difference in case fatality rate between the experimental group and the control group (OR = 1.76, 95% CI (1.29, 2.39), *P*=0.0003, *I*^2^ = 0%, *Z* = 3.58), as shown in Figure 4.

### 3.3. Adverse Events

Review Manager 5.2, a statistical software specialized for meta-analysis, was used to extract and summarize the data, and the analysis statistics were used. For WMD and 95% CI, the *Q* test was first used in the heterogeneity test of included studies. Vascular pseudo-Willebrand factor antigen concentration in the case group and control group was used to compare the results of the analysis. First of all, heterogeneity inspection into the results of the study does not exist between heterogeneity and meta-analysis uses the fixed-effect model. The result shows that the case group vascular pseudo-Willebrand factor antigen concentration was higher than the control group. Obviously, the difference was statistically significant, so there was a statistical difference in adverse events between the experimental group and the control group (OR = 2.38, 95% CI (1.65, 3.45), *P* < 0.001, *I*^2^ = 0%, *Z* = 4.60), as shown in Figure 5.

### 3.4. Incidence of Joint Hemorrhage

Review Manager 5.2, a statistical software specialized for meta-analysis, was used to extract and summarize the data, and the analysis statistics were used. For WMD and 95% CI, the *Q* test was first used in the heterogeneity test of included studies. Vascular pseudo-Willebrand factor antigen concentration in the case group and control group was used to compare the results of the analysis. First of all, heterogeneity inspection into the results of the study does not exist between heterogeneity and meta-analysis uses the fixed-effect model. The result shows that the case group vascular pseudo-Willebrand factor antigen concentration was higher than the control group. Obviously, the difference was statistically significant, so there was a statistical difference in the incidence of joint hemorrhage between the experimental group and the control group (OR = 2.52, 95% CI (1.62, 3.91), *P* < 0.001, *I*^2^ = 0%, *Z* = 4.12), as shown in Figure 6.

### 3.5. Incidence of Subcutaneous Stasis

Review Manager 5.2, a statistical software specialized for meta-analysis, was used to extract and summarize the data, and the analysis statistics were used. For WMD and 95% CI, the *Q* test was first used in the heterogeneity test of included studies. Vascular pseudo-Willebrand factor antigen concentration in the case group and control group was used to compare the results of the analysis. First of all, heterogeneity inspection into the results of the study does not exist between heterogeneity and meta-analysis uses the fixed-effect model. The result shows that the case group vascular pseudo-Willebrand factor antigen concentration was higher than the control group. Obviously, the difference was statistically significant, so there was a statistical difference in the incidence of subcutaneous stasis between the experimental group and the control group (OR = 1.76, 95% CI (1.26, 2.45), *P*=0.0009, *I*^2^ = 5%, *Z* = 3.33), as shown in Figure 7.

### 3.6. Hematoma Volume

Review Manager 5.2, a statistical software specialized for meta-analysis, was used to extract and summarize the data, and the analysis statistics were used. For WMD and 95% CI, the *Q* test was first used in the heterogeneity test of included studies. Vascular pseudo-Willebrand factor antigen concentration in the case group and control group was used to compare the results of the analysis. First of all, heterogeneity inspection into the results of the study does not exist between heterogeneity and meta-analysis uses the fixed-effect model. The result shows that the case group vascular pseudo-Willebrand factor antigen concentration was higher than the control group. Obviously, the difference was statistically significant, so there was a statistical difference in hematoma volume between the experimental group and the control group (OR = 1.78, 95% CI (1.32, 2.40), *P*=0.0001, *I*^2^ = 23%, *Z* = 3.80), as shown in Figure 8.

## 4. Discussion

In this study, DNA methylation in the promoter region of the vWF gene was significantly correlated with the risk of unexplained recurrent hemophilia, indicating that DNA methylation is involved in the occurrence and development of hemophilia.

vWF is a glycoprotein synthesized by vascular endothelial cells and bone marrow megakaryocytes, which plays an important role in both stage 1 and stage 2 hemostasis [23–25]. Lack of vWF will lead to von Willebrand disease (vWD) in patients. vWF can be cleaved by AD-AMTS13 to inactivate it, and thrombin-sensitive protein-1 may be involved in this regulatory process. vWF levels are influenced by a variety of genetic and environmental factors, among which AB blood type has a greater influence. vWF binds platelets GP1b and collagen mainly through A1 and A3 regions [26]. Further study on the mechanism of synthesis, secretion, degradation, and clearance of vWF, as well as the relationship between the structure and function of vWF, will help to find a new way of hemostasis and prevention and treatment of blood thrombolysis [27]. vWF is a glycoprotein synthesized by vascular endothelial cells and bone marrow megakaryocytes, which plays an important role in both stage 1 and stage 2 hemostasis [28]. Lack of vWF will lead to von Willebrand disease, and the overexpression of vWF plays an important role in thrombosis. The mechanism of synthesis, secretion, degradation, and clearance of vWF as well as the relationship between the structure and function of vWF will help to find new ways of hemostasis and prevention and treatment of thrombosis. The vWF gene is located on chromosome 12, with a total length of 178 KB, consisting of 52 exons and 51 introns [29]. There is a pseudogene of vWF (M60676) on chromosome 22, which is highly homologous with the sequence of vWF23 ∼ 34 exons, and vWF cDNA encodes 2813 amino acid primary transcripts [30].

The main binding sites of vWF and collagen are A1 and A3 of vWF. The Al region is mainly involved in the binding of type IV collagen, while the A3 region is mainly involved in the binding of type I and III collagen. In different situations (e.g., different fluid dynamics or extracellular matrix), regions A1 and A3 will play different roles. The three-dimensional structure (crystal X-ray diffraction and nuclear magnetic resonance), plasmon surface resonance, and mutation analysis showed that the binding site of collagen was located in front of the A3 region, and the front and lower parts (such as D979, S1020, and H1023) were the most important [31]. The front and upper parts (e.g., 1975, T977, V997, and E1001) have weaker binding forces. Related factors are secreted into the blood and closely combined with the vWF in the blood to maintain a constant proportion in the plasma [32]. The fluctuation of the human vWF level can also affect the VIII factor level accordingly. The binding of vWF can maintain the stability of Factor VIII and regulate the activity of Factor VIII, mainly by sealing the phospholipid-binding site of Factor VIII, preventing Factor VIII from participating in the formation of the *X* enzyme complex, and preventing Factor V from being inactivated by antigen-presenting cells [33–35]. In vitro experiments showed that vWF was also involved in the formation of VIII heavy/light chain heterodimers, and the lack of vWF would prevent the formation of VIII light chain heterodimers. Epigenetics plays an important role in the regulation of gene expression and genotype characteristics. It is widespread and participates in the occurrence of diseases. Epigenetic phenomena include a variety of molecular mechanisms, such as histone modification, DNA methylation, and small or noncoding RNAs; DNA methylation is an important component of DNA methylation, which plays an important role in many aspects of the body and is heritable [36]. DNA methylation and mRNA coordinate to regulate transcription. Therefore, gene methylation is necessary, and the degree of methylation of clotting factor genes can affect clotting function. Polymorphism of the coagulation factor vWF gene is associated with recurrent hemophilia of unknown cause.

There are some limitations in this study: (1) the number of relevant cases and the number of included cases are small, and there may be a certain publication bias; (2) the number of references included was small, and there was no subgroup analysis for comparison; (3) the study only assessed the effect of treatment at the end of the study but did not assess medium and long-term efficacy; and (4) different patients were included in the study with different complications, and there was certain heterogeneity.

In this study, the methylation rate of CpG1 and CpG2 sites in the promoter region of the coagulation factor vWF gene associated with unknown recurrent hemophilia was significantly increased, and the difference was statistically significant. This suggests that unexplained recurrent hemophilia may be associated with increased DNA methylation in the promoter region of the coagulation factor vWF gene [37]. The mechanism of abnormal methylation of the coagulation factor vWF gene is speculated in this study to be related to the abnormal function of DNA methyltransferase. Whether demethylation can improve the bleeding index of patients with recurrent hemophilia remains to be further explored.

## Figures and Tables

**Figure 1:** Flowchart of the literature screening.

**Figure 2:** Literature quality evaluation chart. (a) Risk of bias graph and (b) risk of bias summary.

**Figure 3:** (a–d) Funnel plot of literature publication bias.

**Figure 4:** Meta-analysis of case fatality rate between the two groups.

**Figure 5:** Meta-analysis of adverse events between the two groups.

**Figure 6:** Meta-analysis of the incidence of joint hemorrhage between the two groups.

**Figure 7:** Meta-analysis of the incidence of subcutaneous stasis between the two groups.

**Figure 8:** Meta-analysis of hematoma volume between the two groups.

**Table 1:** Basic clinical features of 12 kinds of literature were included in our study.

Study	Age	Gender (male) (%)	Result indicators	Experimental group	Control group	NOS score	Research type
Van Moort et al. 2020 [11]	55.71 ± 1.2	41.25	Case fatality rate, adverse events, etc.	42/59	32/59	7	RCT
Neufeld et al. 2018 [12]	57.65 ± 3.4	59.12	Case fatality rate, adverse events, etc.	56/78	45/78	9	RCT
Lalezari et al. 2014 [13]	43.12 ± 4.5	45.72	Case fatality rate, adverse events, etc.	48/63	42/68	8	RCT
Kessler et al. 2011 [14]	17.15 ± 4.5	44.12	Case fatality rate, adverse events, etc.	107/120	89/120	8	RCT
Gill et al. 2015 [15]	42.85 ± 8.4	51.89	Case fatality rate, adverse events, etc.	122/192	105/192	8	RCT
Mannucci et al. 2013 [16]	64.36 ± 1.2	53.45	Case fatality rate, adverse events, etc.	28/32	22/32	7	RCT
Skotnicki et al. 2016 [17]	32.62 ± 2.2	58.10	Case fatality rate, adverse events, etc.	48/65	40/65	9	RCT
Mannucci et al. 1992 [18]	42.61 ± 3.0	48.75	Case fatality rate, adverse events, etc.	15/18	12/18	9	RCT
Nemes et al. 2007 [19]	57.25 ± 4.5	59.23	Case fatality rate, adverse events, etc.	600/623	567/623	7	RCT
Lethagen et al. 2000 [20]	46.22 ± 5.2	56.22	Case fatality rate, adverse events, etc.	25/30	23/30	7	RCT
Peyvandi et al. 2019 [21]	51.35 ± 2.1	43.16	Case fatality rate, adverse events, etc.	48/52	125/172	8	RCT
Tosetto et al. 2000 [22]	51.25 ± 1.1	46.34	Case fatality rate, adverse events, etc.	28/32	21/32	8	RCT

## Data Availability

The simulation experiment data used to support the findings of this study are available from the corresponding author upon request.
